# Preservation of dendritic spine morphology and postsynaptic signaling markers after treatment with solid lipid curcumin particles in the 5xFAD mouse model of Alzheimer’s amyloidosis

This article has been retracted.

**DOI:** 10.1186/s13195-021-00769-9

**Published:** 2021-02-08

**Authors:** Panchanan Maiti, Zackary Bowers, Ali Bourcier-Schultz, Jarod Morse, Gary L. Dunbar

**Affiliations:** 1 Field Neurosciences Institute Laboratory for Restorative Neurology, Central Michigan University, Mt. Pleasant, MI 48859 USA; 2 Program in Neuroscience, Central Michigan University, Mt. Pleasant, MI 48859 USA; 3 Department of Psychology, Central Michigan University, Mt. Pleasant, MI 48859 USA; 4 Field Neurosciences Institute, Ascension St. Mary’s Hospital, Saginaw, MI 48604 USA; 5 College of Health and Human Services, Saginaw Valley State University, Saginaw, MI 48710 USA

**Keywords:** Alzheimer’s disease, Neurodegeneration, Dendritic spine, Synaptic loss, Curcumin, Pre- and postsynaptic proteins

## Abstract

**Background:**

Synaptic failure is one of the principal events associated with cognitive dysfunction in Alzheimer’s disease (AD). Preservation of existing synapses and prevention of synaptic loss are promising strategies to preserve cognitive function in AD patients. As a potent natural anti-oxidant, anti-amyloid, and anti-inflammatory polyphenol, curcumin (Cur) shows great promise as a therapy for AD. However, hydrophobicity of natural Cur limits its solubility, stability, bioavailability, and clinical utility for AD therapy. We have demonstrated that solid lipid curcumin particles (SLCP) have greater therapeutic potential than natural Cur in vitro and in vivo models of AD. In the present study, we have investigated whether SLCP has any preservative role on affected dendritic spines and synaptic markers in 5xFAD mice.

**Methods:**

Six- and 12-month-old 5xFAD and age-matched wild-type mice received oral administration of SLCP (100 mg/kg body weight) or equivalent amounts of vehicle for 2 months. Neuronal morphology, neurodegeneration, and amyloid plaque load were investigated from prefrontal cortex (PFC), entorhinal cortex (EC), CA1, CA3, and the subicular complex (SC). In addition, the dendritic spine density from apical and basal branches was studied by Golgi-Cox stain. Further, synaptic markers, such as synaptophysin, PSD95, Shank, Homer, Drebrin, Kalirin-7, CREB, and phosphorylated CREB (pCREB) were studied using Western blots. Finally, cognitive and motor functions were assessed using open-field, novel object recognition (NOR) and Morris water maze (MWM) tasks after treatment with SLCP.

**Results:**

We observed an increased number of pyknotic and degenerated cells in all these brain areas in 5xFAD mice and SLCP treatment partially protected against those losses. Decrease in dendritic arborization and dendritic spine density from primary, secondary, and tertiary apical and basal branches were observed in PFC, EC, CA1, and CA3 in both 6- and 12-month-old 5xFAD mice, and SLCP treatments partially preserved the normal morphology of these dendritic spines. In addition, pre- and postsynaptic protein markers were also restored by SLCP treatment. Furthermore, SLCP treatment improved NOR and cognitive function in 5xFAD mice.

**Conclusions:**

Overall, these findings indicate that use of SLCP exerts neuroprotective properties by decreasing amyloid plaque burden, preventing neuronal death, and preserving dendritic spine density and synaptic markers in the 5xFAD mice.

**Supplementary Information:**

The online version contains supplementary material available at 10.1186/s13195-021-00769-9.

## Background

Clinical, biochemical, and experimental evidence suggests that accumulation of misfolded amyloid beta protein (Aβ) and neurofibrillary tangles from hyperphosphorylated tau are strongly associated with neurodegeneration in Alzheimer’s disease (AD) [1, 2]. Aggregation of these misfolded proteins in intra- and extracellular spaces increases neuroinflammation, oxidative stress [3, 4], and neuronal death. In general, accumulation of these misfolded amyloid proteins are considered as the main causative agent for synaptic failure and cognitive impairment in AD [5]. Several experimental reports suggest that these misfolded proteins cause synaptic loss, including decreases in dendritic arborization and dendritic spine loss, which are associated with synaptic dysfunction in AD [6–8]. The number of dendritic spine is directly associated with higher cognitive function and their loss is strongly associated with synaptic dysfunction and cognitive impairment in AD [9]. Many researchers have demonstrated that dendritic branches undergo dynamic changes, including a decrease in number, change in size, and alteration in shape in the AD brain, which directly interferes with synaptic structure and plasticity [8]. Many synaptic signaling proteins, such as postsynaptic density protein 95 (PSD95), Shank, Homer, Drebrin, and Kalirin-7, are downregulated in AD [10]. These signaling proteins are related to dendritic spine remodeling or synaptic plasticity. Although loss of dendritic plasticity and decreases in spine density are closely linked with cognitive impairments in AD, the detailed mechanisms for these changes remain uncertain. Several different mechanisms have been proposed, including intracellular and extracellular deposition of diffusible or soluble Aβ oligomers, tau hyperphosphorylation, and microglial activation [11]. Preventive interventions, such as decreasing neuroinflammation or disaggregating misfolded Aβ and tau tangles are some of the proposed options to prevent neurodegeneration. Therefore, putting emphasis on preservation of existing synapses and reduction of synaptic loss have become major strategies for preserving the cognitive function in AD.

Given that anti-oxidant, anti-inflammatory, and anti-amyloid agents, along with reducing toxicity, would be optimal goals for AD therapy [12, 13]. Therefore, removal of amyloid aggregates, activating Aβ degrading enzymes, boosting immunity or activating protein-clearance pathways could be the viable strategies to prevent AD pathogenesis. Over the past few decades, several natural, as well as recombinant or synthesized anti-amyloid and anti-inflammatory compounds, have been explored as ways to prevent or treat AD. However, many of these approaches are fraught with toxic side effects when tested in vivo. Beyond the limited FDA-approved drugs, other methods, such as β-sheet blockers, anti-amyloid compounds, and immunotherapies, have been developed to counter AD-induced pathology [14, 15].

Because of its unique and ideal physical, chemical, and biological properties, as well as its potent anti-oxidant and anti-inflammatory capabilities, curcumin (Cur), a natural, active polyphenol, has been extensively investigated by several laboratories, including our own, as a means of preventing and treating AD [16–21]. Curcumin is the most active compound in turmeric and it is a popular spice and dietary supplement used world-wide, especially in South Asian countries. Derived from the root of the herb *Curcuma longa* L. (family: Zingiberaceae) [22], Cur can cross the blood brain barrier (BBB), penetrate into brains, and protect neurons from Aβ-induced neuronal death [16, 19, 21]. Ma and colleagues [23, 24] have demonstrated that Cur suppresses soluble tau dimers and protects key molecular chaperones, as well as reduces synaptic loss and behavioral deficits in aged transgenic mouse models of AD. Recently, McClure and colleague [25, 26] reported that aerosol delivery of Cur reduced Aβ deposition and improved cognitive performance in a transgenic model of AD. Similarly, He and colleagues reported that Cur improved the structure and function of the synapses by regulating the synapse-related proteins PSD95 and Shank1, in APPswe/PS1dE9 mice [27].

However, natural Cur has poor solubility in most of the body fluids, accounting for its low bioavailability [28]. Recently, several formulations were developed to increase the bioavailability of Cur [21, 24]. During the last few years, our laboratory has been exploring the efficacy of solid lipid curcumin particles (SLCPs) to reduce the dysfunction observed in neurodegenerative diseases [18–21, 29–32]. We also demonstrated that acute treatment of SLCP provides more anti-amyloid, anti-inflammatory, and neuroprotective effects than does natural Cur in the 5xFAD mouse model of AD [29]. In addition, our comparative studies showed that SLCP has greater neuroprotection and Aβ aggregation inhibition than does natural Cur in cultured mouse neuroblastomas after exposure to Aβ42 [19]. We also reported that SLCP has greater affinity to bind to Aβ and inhibits their aggregation more than natural Cur in vitro and in the 5xFAD mice [21]. Although Cur treatment improved cognitive function in different animal models of AD, the molecular mechanisms of these cognitive and behavioral improvements remain to be elucidated. In an effort to explore the mechanisms of Cur-induced therapeutic efficacy, we tested whether Cur preserves synaptic plasticity and function by preventing dendritic spine loss and by preserving synaptic markers.

To do this, we designed our study to investigate the effects of SLCP on Aβ plaque loads, neurodegeneration, dendritic arborization, spine density, pre- and postsynaptic markers, and behavioral outcomes in 5xFAD mice. Our results suggest that the SLCP decreases amyloid plaques and neuronal death, prevents dendritic spine loss, and preserves pre- and postsynaptic markers, along with partially improving behavioral outcomes in the 5xFAD mouse model of AD.

## Materials and methods

### Chemicals

Ammonia solution, sodium thiosulfate, Trizma-base, glycine, protease cocktail, cresyl violet stain, normal goat serum, Triton-X100, paraformaldehyde, and curcumin were purchased from Sigma (St. Louis, MO). Mercury chloride, potassium dichromate and potassium chromate, and methanol were procured from Fisher Scientific (Hampton, NH). Fluoro-jade C and polyvinylidene difluoride (PVDF) membranes were purchased from EMD-Millipore (Burlington, MA). DePeX mounting media was purchased from BDH (Radnor, PA). 4′,6-Diamidino-2-phenylindole (DAPI) was from IHC-world (San Diego, CA). BCA Kit was purchased from Thermo Fisher Scientific (Waltham, MA). Non-fat dry milk powder was obtained from RPI-Research Product (Mount Prospect, IL). Sodium deoxycholate was bought from Alfa Aesar (Haverhill, MA). Nonidet-P40 was obtained from US Biological (Salem, MA). Fatal-Plus anesthetic solution was bought from Drugs.com (https://www.drugs.com/vet/fatal-plus-solution.html). Solid lipid curcumin particles (SLCP), which contain 26% Cur, were gifted from the Verdure Sciences (Noblesville, IN). This formulation contains high-purity, long-chain phospholipid bilayer and a long-chain fatty acid solid lipid core, which coates curcumin. The SLCP formulation has been characterized by our laboratory and others with in vitro [21], and in animal models [23, 30–32], as well as in clinical trials of AD [33]. Detailed information for all the antibodies used in this study are documented in Table 1.

**Table 1:** Different antibodies and their sources used for this study

Antibodies	Source	Type	Company	Catalog no.	Address
Synaptophysin	Rabbit	Monoclonal	Cell signaling Technology	5461S	Danvers, MA
PSD95	Mouse	Monoclonal	Santa Cruz Biotech	sc-32290	Santa Cruz, CA
Shank1/2/3	Mouse	Monoclonal	Santa Cruz Biotech	4272S	Santa Cruz, CA
Homer	Rabbit	Polyclonal	Cell Signaling Technology	8231S	Danvers, MA
Drebrin	Rabbit	Polyclonal	Cell signaling Technology	12243S	Danvers, MA
Kalirin	Goat	Polyclonal	Abcam	Ab52012	Cambridge, MA
CREB	Rabbit	Monoclonal	Cell signaling Technology	9197S	Danvers, MA
pCREB (Ser133)	Rabbit	Monoclonal	Cell signaling Technology	9198S	Danvers, MA
GAPDH	Rabbit	Monoclonal	Cell signaling Technology	5174S	Danvers, MA
β-tubulin	Rabbit	Monoclonal	Cell signaling Technology	2128S	Danvers, MA
6E10	Mouse	Monoclonal	Bio-Legend	SIG 39320	San Diego, CA
2^o^Ab antibodies			Santa Cruz Biotech		San Diego, CA

### Dot blot assay

To compare the anti-amyloid potency, such as inhibition of Aβ42 aggregation after treatment with SLCP and natural Cur, the dot blot assay was performed, as described previously [34, 35]. Briefly, Aβ42 peptide was dissolved in hexafluoro isopropanol (HFIP), mixed for 1 min and allowed to solubilize for 30 min at room temperature, and then the HFIP was evaporated under laminar hood to make a thin film of peptide layer. The thin peptide film was stored at − 20 °C until use. The peptide was dissolved in 60-mM NaOH (final concentration was 6 mM) and diluted with Tris-buffered saline (TBS; 0.1 M, pH 7.4) with 0.025% sodium azide. The final peptide concentration was 10 μM. Approximately, 50 μL of peptide solution (10 μM) was taken in a 200-μL Eppendorf tube and incubated, with or without different concentrations of Cur or SLCP (in μM: 100, 10, 1, 0.1, 0.01, 0.001), for 8, 24, 48, and 72 h at 37 °C, with gentle shaking (200 rpm). After incubation, about 10 μL of peptide solution was spotted on PVDF membrane (Bio-Rad, CA, USA) and dried for 30 min at room temperature. The membrane was blocked with 5% non-fat milk in TBS-Tween-20 (TBS-T) at room temperature for 1 h and incubated with A11, OC, and 6E10 (1: 1000) in 5% non-fat milk powder in TBS-T overnight at 4 °C. After washing, the membrane was probed with anti-rabbit horseradish-peroxidase (HRP), conjugated secondary antibody solution (1: 25,000, Santa Cruz Biotech, CA, USA) for 1 h at room temperature. The blot was developed with ImmobilonTM Western Chemiluminescent HRP-substrate (Thermo Fisher Scientific). The dot blots were scanned using gel documentation system (Bio-Rad, CA, USA), and the optical density of each dot was measured using ImageJ software (http://imagej.nih.gov).

### Animals

Six-month-old and 1-year-old B6SJL-Tg (APPSwFlLon, PSEN1*M146L*L286V, 1136799Vas/J; Jackson Laboratory, stock no: 34840-JAX/5xFAD) and age-matched wild-type, male and female mice were used in this study. The 5xFAD mice overexpressed human APP and PS1 with five familial AD mutations, including three mutations in the APP gene [Swedish (K670N, M671L), Florida (I716V), and London (V717I)] and two in the PS1 gene (M146L and L286V) [36, 37]. A detailed pathology of 5xFAD mice was described by many investigators, previously [21, 38–40]. All mice were housed at 22 °C at Saginaw Valley State University neuroscience vivarium under a 12-h light/12-h dark, reverse-light cycle with *ad libitum* access of food and water. Transgenic characteristics of all 5xFAD mice were confirmed by genotyping at 3 weeks of age using polymerase chain reaction (PCR). *This study was carried out in strict accordance with the protocols* approved by the Institutional Animal Care and Use Committee *of* the Saginaw Valley State University (IACUC no- 1513829-1). *All surgeries were performed using Fatal-plus as  anesthesia (1 ml/4.54 kg body weight), and all efforts were made to minimize animal discomfort.*

### Solid lipid curcumin particle (SLCP) treatment

A total of 96 mice 5xFAD and age-matched wild-type (WT) mice at 6 or 12 months of age were administered SLCP (100 mg/kg body weight), or equivalent volumes of vehicle (0.5% methylcellulose), orally, every other day for 2 months. The dose selection was based on our previous studies [21]. The mice were randomly divided into eight groups shown in Table 2. The SLCP was dissolved in 0.5% methylcellulose in PBS (0.1 M, pH 7.4). Treatments were initiated 4 days after baseline behavioral tests and continued for 60 days. The same volume of vehicle (0.5% methylcellulose, dissolved in 0.1 M PBS, at pH 7.4) was administered to the vehicle groups as summarized in Table 2.

**Table 2:** Experimental groups and timeline. Distribution of a total of 96 mice 6- and 12-month-old 5xFAD and age-matched WT mice for each procedural group. All mice were treated orally with SLCP (100 mg/kg BW) every other day for 2 months. *IF* immunofluorescent, *GC* Golgi-Cox, *FJC* fluoro-jade C, *m* month

Groups	Group (m)	Behavior	CV stain	GC stain	Histochemistry	Western blot
WT + vehicle	6	12 (M = 4, F = 2)	3 (M = 2, F = 1)	6 (M = 4, F = 2)	3 (M = 2, F = 1)	3 (M = 2, F = 1)
5xFAD + vehicle	6	12 (M = 4, F = 2)	3 (M = 1, F = 2)	3 (M = 1, F = 2)	3 (M = 2, F = 1)	3 (M = 2, F = 1)
5xFAD + SLCP	6	12 (M = 2, F = 4)	3 (M = 2, F = 1)	3 (M = 2, F = 1)	3 (M = 1, F = 2)	3 (F = 3)
WT + SLCP	6	12 (M = 4)	3 (M = 1, F = 2)	6 (M = 3, F = 3)	3 (M = 1, F = 2)	3 (M = 2, F = 1)
WT + vehicle	12	11 (M = 6, F = 5)	3 (M = 2, F = 1)	3 (M = 2, F = 1)	3 (M = 2, F = 1)	3 (M = 1, F = 2)
5xFAD + vehicle	12	10 (M = 6, F = 4)	3 (M = 2, F = 1)	6 (M = 2, F = 4)	3 (M = 2, F = 1)	3 (M = 2, F = 1)
5xFAD + SLCP	12	11 (M = 7, F = 4)	3 (M = 1, F = 2)	3 (M = 1, F = 2)	3 (M = 1, F = 2)	3 (M = 1, F = 2)
WT + vehicle	12	10 ((M = 6, F = 4)	3 (M = 2, F = 1)	6 (M = 2, F = 1)	3 (M = 2, F = 1)	3 (M = 1, F = 2)

## Behavioral assays

### Open field test

Baseline measures in the open-field (OF) test was obtained at “day 0,” treatments, and prior to OF testing began at “day 66” post-treatment (see S1). The OF test was used to measure spontaneous locomotor activity, including exploratory behavior, as described previously [41, 42]. The OF test apparatus consisted of a Plexiglas box (41 cm × 41 cm × 30 cm high; San Diego Instruments, San Diego, CA) with grids of infrared beams spaced 2.5 cm from the OF floor (used to measure horizontal activity) and 7.5 cm from the OF floor (used to measure vertical, or rearing activity) around the sides of the OF. Each of the infrared grids consisted of 16 photobeams in each direction (16 × 16) in which the location of the mouse could be tracked each time the infrared beams in the area was blocked by movements of the mouse. The automated software was connected to the system used to measure the overall movement of the mice, as indicated by the number of breaks in the gridded infrared beam system. For OF testing, each mouse was placed into the chamber and allowed to explore for 30 min. Total resting time, total distance traveled, and velocity of movement were measured throughout the entire time. In addition, counts of fecal boli were taken as a potential indicator of anxiety.

### Novel object recognition

The novel object recognition (NOR) test is one of the most commonly used behavioral tests for investigating various aspects of learning and memory in mice. The detailed protocol was described by Leuptow and colleagues [41, 43]. The NOR was performed in a gray polyvinyl plastic testing box (40 cm × 40 cm × 40 cm). The test consists of two phases: habituation and acquisition. In habituation, the mice were allowed to familiarize themselves with the NOR environment for 10 min. The next day, the mice were given 10 min to explore two identical objects, which were placed near the center of the box at 14.75 cm from the walls and 25 cm apart from each other. For this purpose, we placed two circular, white, odorless polypropylene objects (3 cm × 2 cm), which served as familiar objects (FOs). After 10 min of exploration with the FOs, the mouse was returned to its home cage for 5 min, during which time one of the FOs was replaced with a new, white, rectangular, odorless object (3 cm × 2 cm), which served as novel object (NO) and the mice were then allowed to explore these objects for another 10 min. The boxes and the objects were cleaned between each trial with 70% ethanol, which was allowed to dry prior to the next trial. The entire experiment was video-recorded using an overhead camera, attached with Any-Maze software (Columbus, OH). Using this automated software, the exploration time of novel object (TN) contact and exploration time the familiar object  (TF) contact was measured. The exploratory index was measured by using the following equation: (TN − TF). The discrimination index (DI) was calculated with the following equation: (TN − TF)/(TN + TF) × 100. The NOR was conducted on days 2–4 prior to treatment and on days 67–69 after the start of treatment.

### Morris water maze (MWM)

Morris water maze (MWM) task was used to assess spatial memory, as described previously [41, 44–46]. In this task, mice are required to learn the spatial location of the hidden platform in a circular pool (180 cm in diameter and 153 cm in height) filled with water to a depth of 90 cm and kept at 20–25 °C. The water was made opaque by the addition of non-toxic white paint to obscure a rectangular transparent platform (10 cm × 10 cm), which was placed 1.5 cm below the surface of the water, in the Southeast (SE) quadrant of the tank. The MWM tank was kept in a 3.6 × 3.3 m room, with illumination provided by four overhead 200-watt mercury lamps. The foreheads of the mice were marked using black permamarker to facilitate tracking their swim path. The MWM tank was divided into four quadrants: Southeast (SE), Northeast (NE), Northwest (NW), and Southwest (SW). The platform was kept in the center of the SE quadrant. An overhead camera and computer-assisted tracking system (Any-Maze, USA) recorded the movement of the mouse in the maze, which enabled measurements of latency (time taken to reach the hidden platform) and path length (distance swam by mice) to find the hidden platform. All trials in each experiment were performed between 900 and 1200 h. All mice were given four trials per day, with an inter-trial interval of 10 min. The trials were carried out over 5 days (20 sessions). A trial consisted of gently placing the mouse by hand into the water, facing the wall of the pool at one of four equally spaced starting points (N, S, E, and W) and allowing the mouse to swim for 60 s. One day prior to the first day of testing, the mice were given four habituation trials and if they did not find the hidden platform within the MWM for 60 s, they were guided by hand to the platform and were allowed to rest on it for 30 s. The procedure was followed during testing, except a different starting point was used on each of the four trials with the order determined randomly. After finding or being guided to the platform, the mice were allowed to remain on it for 30 s, after which they were removed and gently towel-dried, before being placed back into their home cages. The dependent measure for this task included the latency and pathlength to find the platform. Average speed of the animals (distance/time) was also calculated. The MWM experiment was conducted on days 70–75 following the start of treatment.

One day after the last training trial, all mice were placed in the MWM tank facing the “N” starting point and allowed to swim for 60 s. The number of entries, total time, and distance swum by every mouse in each quadrant was recorded using an automated behavioral tracking software (Any-Maze, Columbus instruments, USA).

## Tissue processing

Mice used for histological studies are shown in Table 2. For histology and immunofluorescent studies, the mice were deeply anesthetized with an overdose of Fatal-Plus (0.22 ml/kg of body weight, i.p.) and transcardially perfused with 0.1 M cold PBS at pH 7.4, followed by a 4% paraformaldehyde (diluted in 0.1 M PBS at pH 7.4) fixation solution. The brains were extracted from the cranial vault and post-fixed with the 4% paraformaldehyde and stored at 4 °C until their use. For Golgi-Cox (GC) staining, mice were cervically dislocated, and their brains were extracted and dropped into GC solution. Similarly, for Western blot sample preparation, mice were cervically dislocated, their brains were extracted, and their hippocampi and cortices were dissected out of 4 °C and stored at − 80 °C, until use.

### Neuronal morphology by cresyl violet staining

One of the aims of this study was to investigate whether SLCP can reduce abnormal neuronal morphology in the 5xFAD mice, especially in prefrontal cortex (PFC), hippocampal subfields, and entorhinal cortex (EC). Briefly, the brains from all groups were dehydrated with graded alcohol and processed with paraffin embedding and were sectioned at 5 μm using a rotary microtome, before being stained with 0.1% cresyl violet, as described previously [45, 47, 48]. The sections were washed, dehydrated with graded alcohol, cleared, mounted, and cover-slipped using DePex (BDH, Batavia, IL). Photomicrographs were taken using a compound light microscope (Olympus, Japan) with a  40x objective (total magnification of 400x). The number of pyknotic cells were counted manually using ImageJ software (http://imagej.nih.gov/ij) and were expressed as number of pyknotic cells per 100 μm^2^ area sampled. A minimum of 5 different sections from each brain area, each with 10 different fields, were used for counting the number of pyknotic cells in each group.

### Fluoro-jade C staining

To investigate the number of degenerated neurons in 5xFAD mice and to determine whether SLCP treatment prevented an increase in these numbers, brain sections were stained with fluoro-jade C (FJC), a poly-anionic fluorescence dye which specifically binds to degenerating neurons. The staining method was adapted from Schmued and colleague [49], with some modifications [47]. Briefly, the perfused and post-fixed brains were transferred to the graded sucrose solutions (10%, 20%, and 30%, dissolved in 0.1 M PBS, pH 7.4), and coronal sections (40 μm) were made on a cryostat (Leica, Germany). The coronal sections (40 μm thick) were washed with PBS for 5 min and then washed in distilled water for 1 min. The sections were treated with freshly prepared 0.06% potassium permanganate solution (dissolved in distilled water) and placed on a shaker for 20 min. Then the sections were washed with distilled water and stained with FJC (0.001% in distilled water) for 30 min at room temperature in the dark, while undergoing gentle shaking. After staining, the sections were washed 3 times with distilled water for 1 min each before being air dried. The sections were cleared with xylene and then mounted in DePex. The image was taken with a fluorescence microscope (Leica, Germany) using appropriate excitation/emission filters. A bright green fluorescence signal indicated degenerated neurons, which were counted manually using ImageJ software (http://imagej.nih.gov/ij) and expressed as number of FJC-positive neurons per microscopic field.

### Amyloid β-plaques staining

To investigate the effects of SLCP on Aβ plaque burden, coronal (40-μm) sections were obtained from the brains of 5xFAD and WT mice using a cryostat. These sections were stained with 6E10 and curcumin, which specifically binds with Aβ plaques [21, 50]. The number of Aβ plaques was counted in PFC, CA1, and CA3 areas. Cur was used to label Aβ plaques, because it labels plaques as efficiently as Aβ-specific antibody as described previously by us [21]. Using ImageJ software (http://imagej.nih.gov/ij), the total area of each image was measured and the numbers of Aβ plaques were counted manually in PFC, CA1, CA3, DG, subicular complex, and EC area and expressed as the number of Aβ plaques per 100 μm^2^ area. Only clearly visible, large fluorescent signals were counted as Aβ plaques. A minimum of 10 serial sections, with 20–30 different fields were counted for Aβ plaques, and the mean from each group (*n* = 3/group) was calculated from the counts by two researchers, who were blinded to the group identity of the specimens sampled [41].

### Golgi-Cox staining

Dendritic arborization and number of dendritic spines were studied by Golgi-Cox (GC) stain, as described previously [34, 44, 47]. Briefly, equal volumes of 5% potassium dichromate (solution A) and 5% of mercuric chloride (solution B) were mixed (dissolved in double-distilled water) in a glass beaker (AB mixture). In a separate glass beaker, four volumes of 5% solution of potassium chromate (solution C) was diluted with ten volumes of distilled water. Then the AB mixture was slowly mixed with solution C and was stirred in the dark for 1 h using a magnetic stirrer. The solution was then stored in a glass-stoppered bottle and kept in the dark at room temperature for 5 days. Using Whatman filter paper, the GC solution was then filtered and stored in a large brown glass bottle, until needed. The mice were euthanized via 0.22 ml/kg of Fetal-Plus, and their brains were extracted and placed into vials containing GC solution (ten volumes of brain weight), and then kept in the dark for 2 days, at room temperature. After 2 days, freshly prepared GC solution was exchanged, and the brains were allowed to incubate for 2 weeks in dark at room temperature. After 2 weeks of incubation, the GC solution was removed, and the excess GC solution was blotted using tissue paper and the brains were immersed in 30% sucrose solution (dissolved in distilled water) and stored in refrigerator, until they sank. Using vibratome (1000 Plus, Pelco 102, Te Pella Inc., Redding, CA), 150-μm-thick coronal sections were prepared and collected in 6% sucrose solution (vibratome reservoir with the 6% sucrose solution). Each coronal section was then collected on a 0.5% gelatin-coated slide and stored at room temperature in a humidified chamber for at least 7 days, before staining. The mounted sections were then washed with double-distilled water, two times, 2 min each, to remove traces of the impregnating GC solution. Then the sections were immersed in 75% ammonia solution for 10 min in the dark at room temperature, followed by 6 washings of 5 min each with double-distilled water. The sections were then treated with 1% sodium thiosulfate to fix the stain for 10 min at room temperature, in the dark, and washed with double-distilled water, six times, for 5 min each. Then the sections were dehydrated with graded alcohol solutions for 4 min each and processed through two changes of 100% alcohol, 4 min each, cleared with xylene, three times, at 4 min each, and the sections were then left in fresh xylene for 1–2 h, in the dark. Finally, the slides were cover-slipped with DPX/Permount (BDH) and allowed to dry under a fume hood for 3 days before microscopic examination. Individual neurons were imaged using an Olympus microscope at × 40 objectives (BX51, Olympus, Japan), whereas dendritic spines were imaged using × 100, using oil-immersion objectives.

#### Quantification of dendritic spine density

About 40 primary, secondary, and tertiary branches of apical and basal dendrites from 15 to 20 different randomly selected neurons were imaged from PFC, entorhinal cortex, CA1, and CA3 areas using a × 100 objectives (Olympus, total magnification × 1000), as described previously [44]. The number of dendritic spines were counted using ImageJ software (https://imagej.nih.gov/ij/download.html) and expressed as number/100 μm of dendritic length. The counting of dendritic spine density was taken from a dendritic branch which was at least 100 μm long and within a single plane of focus. In addition, counting was performed only from 2- to 3-μm-thick primary branches, 1–2-μm-thick secondary branches, and ≤ 1-μm-thick tertiary branches in order to both minimize the number of spines hidden by the dendritic shaft and to ensure that the number of hidden spines was proportional across all measurements. Double-headed spines were counted as two spines. Individual counts were made by two researchers who were blinded to the group identity of the samples, and the average value was expressed as the number of spine/100 μm of dendritic length [44].

### Immunohistochemistry of synaptic markers

Free floating 40-μm-thick coronal sections were blocked with 10% normal goat serum (NGS) in Tris-buffered saline with 0.5% Triton-X100 (TBS-T) and incubated for 1 h in room temperature. Then sections were then incubated on a shaker, overnight at 4 °C with synaptophysin and PSD95 (rabbit monoclonal, 1:500, Table 3) with 10% NGS in TBS-T. The next day, the sections were washed with TBS-T for 15 min, for three times, and incubated with anti-rabbit secondary antibody (1: 1000), tagged with Alexa fluorophore 595, and incubated for 1 h at room temperature on a shaker in the dark. After three more washings with PBS, the tissue was counter-stained with DAPI for 10 min and washed with distilled water. Then the sections were mounted on poly-L-lysine-coated slides and dehydrated in ascending alcohol series (50%, 70%, and 100%), cleared with xylene and cover-slipped with Fluor-mount media. The signal was detected using a fluorescent microscope (Leica, Germany) with appropriate excitation/emission filters.

**Table 3:** Percentage of inhibition of Aβ42 aggregation by Cur or SLCP in comparison to untreated group, *p < 0.05, **p < 0.01, relative to untreated Aβ42

	6-E10 antibodies				OC antibodies				A11 antibody	
Duration	24 h		48 h		24 h		48 h		8 h	
Treatment Groups	Aβ42+ Cur	Aβ42+ SLCP	Aβ42+ Cur	Aβ42+ SLCP	Aβ42+ Cur	Aβ42+ SLCP	Aβ42+ Cur	Aβ42+ SLCP	Aβ42+ Cur	Aβ42+ SLCP
1 μM	64.54	48.34*	26.25	51.68**	16.99	41.04**	18.95	37.11*	24.20	43.75*
100 nM	71.99	48.44**	31.21	58.69**	21.64	30.59	60.81	36.45*	7.63	48.37**
10 nM	63.96	59.76	18.38	65.70**	27.54	35.15	105.15	33.29*	17.59	53.68**
1 nM	65.05	55.82*	37.34	65.00**	23.07	38.70*	− 73.09	56.82**	22.37	46.74*

## Western blots

After 2 months of treatment, the mice were sacrificed by cervical dislocation, and the hippocampus and cortex were dissected over ice. The tissue was homogenized using tissue homogenizer (Fisher Scientific, Hampton, NH) with ice-cold radio immune precipitation assay (RIPA) buffer and a protease inhibitor cocktail (Sigma, Catalog no: P8340-5ML), as described previously [18, 35, 48]. We were interested to investigate proteins from both membrane-bound and cytosolic fraction together and the RIPA buffer which extracts both membrane-bound, as well as cytosolic proteins together. After centrifugation of tissue homogenate at 13,300 rpm for 20 min at 4 °C, the supernatant was collected, aliquoted with 20 μL in each PCR tube, and stored at − 80 °C until needed. Total protein was quantified with the BCA protein assay kit. The protein samples were run in SDS-PAGE Tris-glycine gel (4–20%). Proteins were transferred overnight to PVDF membranes. The membranes were blocked with 5% non-fat milk for 1 h at room temperature and then were incubated with primary antibodies (1:1000, Table 1) at 4 °C overnight on a shaker. The membranes were washed with fresh Tris-buffered saline and Tween 20 (TBS-T), 3 times, and incubated with the appropriate secondary antibody (1:20,000 dilution) for 1 h at room temperature. The signal was developed by chemiluminescence reagents and detected by gel documentation system (Bio-Rad, Hercules, CA).

## Statistical analyses

The behavioral and morphometric data were expressed as mean ± SEM. All data were analyzed using one-way analysis of variance (ANOVA) with Tukey HSD (honestly significant difference) post hoc tests being conducted when appropriate. Statistical analyses were conducted using the online software available at https://astatsa.com/OneWay_Anova_with_TukeyHSD/. A probability value ≤ 0.05 was considered statistically significant.

## Results

### SLCP inhibited Aβ42 aggregation more effectively than Cur in vitro

Aβ42 aggregation inhibition was monitored using 6E10, A11, and OC antibodies after treatment with Cur and SLCP for different time points. Aβ42 aggregation was inhibited significantly after 24–72 h of incubation with Cur and or SLCP, as shown by probing with 6E10 (S2A-F). Similarly, Aβ42 oligomers (S2G & H) and fibril formation (S2I-L) were significantly inhibited by both Cur and SLCP. Lower concentrations of both Cur and SLCP (1–10 nM) inhibited Aβ42 more effectively than higher concentrations (10–100 μM). In addition, SLCP showed significantly more inhibition of Aβ42 aggregation than Cur treatment (S1). Below is the comparative Aβ42 aggregation inhibition by Cur and or SLCP in comparison to untreated group (Table 3).

### Body weights

There was no significant change in animal weight among the groups in either the 6- or 12-month-old groups of mice during the course of treatments (data not shown).

### Open field test

Open-field testing was used to assess spontaneous locomotor activity levels and anxiety in 5xFAD mice, before and after treatment with SLCP. Although both the 6- and 12-month-old 5xFAD mice were active before and after the treatment began this hyperactivity dissipated in the SLCP-treated mice in both age groups during the re-test (S3E & F). Increased anxiety may have contributed to the initial hyperactivity, as counts of fecal boli from each group of mice revealed a significant increase for 5xFAD mice, in comparison to WT in pre-treated mice at both 6- and 12-months of age (S3E & F).

### Novel objective recognition

The novel object recognition (NOR) test was used to investigate the memory abilities of mice for familiar objects. We observed that 12-month-old, but not 6-month-old 5xFAD mice spent significantly less time exploring the novel object than WT mice, but these recognition memory deficits were prevented by SLCP treatments (S4A). The exploration index revealed a significant decrease for the 12- but not the 6-month-old 5xFAD mice (S4B), while the discrimination index indicated that 5xFAD mice in both the 6-and 12-month-old groups was significantly reduced and SCLP treatments prevented this loss in all cases (S4C).

### Morris water maze (MWM)

The MWM task was used to explore whether SLCP treatment preserves spatial memory abilities in 5xFAD mice. The learning curve for 5 days of MWM training showed that 6- and 12-month-oldvehicle-treated 5xFAD mice took significantly longer time to reach the platform on days 4 and 5 in comparison to WT + vehicle, 5xFAD + SLCP, and WT + SLCP-treated mice (Fig. 1a-b). Similarly, the 12-month-old, but not the 6-month-old vehicle-treated 5xFAD mice swam significantly farther to reach the platform in comparison to all other groups of mice at both 6- and 12- months of age (Fig. 1c, d). Because no significant changes in overall swim speed (cm/s) were observed among any of the 6- and 12-month-old groups of mice (data not shown), the differences observed in length of swim path and latency to find the hidden platform reflect mnemonic changes, rather than motoric ones.

**Fig. 1:** SLCP treatment improved learning and memory in 5xFAD mice. Six- and twelve-month-old 5xFAD and age-matched control animals were tested on the Morris water maze (MWM) task for 5 days, following 2 months of treatment with SLCP (100 mg/kg) or vehicle. The escape latency (**a, b**) and path length (**c, d**) were significantly longer in the case of 12-month-old group of 5xFAD mice in comparison to 5xFAD mice treated with SLCP and WT mice treated with vehicle. **e–h** After 5 days of training in MWM, all mice were given a 60-s probe trial and the latency to first enter to the target quadrant (**e**), mean distance from the target (previous location of platform) (F), mean number of entries in target quadrant (G) and the time spent in target quadrant (**h**) were measured. There was an increase in latency of first entry to the target quadrant (**e**) for vehicle-treated 5xFAD mice, whereas SLCP treatment prevented this increase. Mean distance from the platform was significantly increased in both 6- and 12-month-old 5xFAD mice (**f**), but this was prevented by treatment with SLCP. Mean number of entries (**g**) was not significantly different among all the animal groups. Time spent in the target quadrant was decreased for the 6-, but not the 12-month-old 5xFAD mice (**h**), and this deficit was mitigated by the SLCP treatment. *p < 0.05, **p < 0.01, and ***p < 0.001 in comparison to WT + Vehicle, 5xFAD + SLCP, and WT + SLCP

#### Probe trial data

Latency of first entry (Fig. 1e) and mean distance from the quadrant (Fig. 1f) which previously contained the platform (i.e., the target quadrant) was significantly reduced for both the 6- and 12-month-old 5xFAD mice in comparison with their age-matched WT + vehicle-treated and SLCP+5xFAD mice. However, no significant between-group differences for mean number of entries to the target quadrant for either age group (Fig. 1g) or time spent in the target quadrant (Fig. 1h) for the 12-month-old mice were observed. However, 6-month-old vehicle-treated 5xFAD mice spent less time in the target quadrant and both the 6- (Fig. 1h) and 12-month-old vehicle-treated 5xFAD mice averaged more distance from the target quadrant (Fig. 1f) than did those treated with SLCP.

### SLCP reduced pyknotic cells and neurodegeneration in different brain areas of 5xFAD mice after treatment with SLCP

One of the aims of this study was to investigate whether a chronic 2-month treatment of SLCP protects the neuronal morphology in cortical and hippocampal subfields. Paraffin-embedded tissue sections were stained with 0.1% cresyl violet and the number of pyknotic or tangle-like neurons was counted within the pyramidal layers of the PFC, EC and the CA1, and CA3 subfields of hippocampus. In the case of PFC and EC, we observed a significant increase in the percentage of pyknotic cells in 5xFAD mice, whereas treatment with SLCP significantly mitigated the percentage of pyknotic cells in 5xFAD mice when compared to 5xFAD + vehicle-treated mice (Fig. 2a–c). Similarly, a significant increase in percentage of pyknotic cells were observed in the CA1 and CA3 subfields of hippocampus in 5xFAD mice in both 6- and 12-month-old mice, whereas SLCP treatment prevented this (Fig. 2a, d, e). Similar finding was observed in the entorhinal cortex (data not shown). The number of damaged were more prevalent in the case of 12-month-old mice, relative to 6-month-old group in all three brain regions. Similarly, we found more pyknotic cells in the CA3 area (Fig. 2e) than in other areas for both the 6- and 12-month-old 5xFAD mice (Table 4).

**Fig. 2:** SLCP treatment decreased pyknotic cells and degenerated neurons in PFC and hippocampus and entorhinal cortex of 5xFAD mice. Six and twelve-month-old 5xFAD and age-matched control mice were treated with SLCP (100 mg/kg) or vehicle for 2 months at which they were euthanized, and their brains were perfused with 4% paraformaldehyde. The brains were embedded in paraffin and cut on a rotary microtome into 5-μm coronal sections which were stained with 0.1% cresyl violet. Images were taken through compound light microscope using  40x objectives (total magnification  400x). There was a significant increase in the percentage of pyknotic cells in the PFC (**a, b**), and in the EC (**a, c**) and CA1 (**a, d**) and CA3 (**a, e**) areas of hippocampus of the vehicle-treated 5xFAD mice, but these increases were mitigated by SLCP treatments. **f** Image with the white arrow indicating normal and the red arrow indicating pyknotic neurons. **h–k** Forty-micron coronal sections were stained with fluoro-jade C (FJC) solution (0.0001%). Images were taken using a fluorescent microscope with a  20x objective (total magnification = × 200). There were significant increases in the number of FJCs in PFC, and in the CA1 and CA3 areas of the hippocampus in the vehicle-treated 5xFAD mice in both 6- (**h, i**) and 12-month-old (**j, k**) mice, whereas SLCP treatment prevented these increases. **g** Yellow arrow indicating FJB positive degenerated neuron. *p < 0.05, **p < 0.01 in comparison to WT + vehicle, 5xFAD + SLCP, and WT + SLCP. Red arrows indicate FJC-positive degenerated neurons. Large fluorescent signals are Aβ plaques. Scale bar = 100 μm and is applicable to all images

**Table 4:** Percentage pyknotic cells in treated and untreated 5xFAD and age-matched WT mice. *p < 0.05; **p < 0.01 compared to WT + vehicle and WT + SLCP. ↓ decrease, *m* month

Groups	Pyknotic cells							
	PFC		CA1		CA3		EC	
	6 m	12 m	6 m	12 m	6 m	12 m	6 m	12 m
5xFAD + vehicle	22.98**	31.91**	22.14**	36.12**	29.16**	44.89**	20.73	29.79
5xFAD + SLCP	14.15*	18.41*	9.86**	18.27**	22.38**	24.34**	13.17*	15.13*
% ↓ pyknotic cells by SLCP treatment	38.45	42.29	55.45	49.40	23.25	45.76	36.48	49.19
5xFAD + vehicle	36.27	45.89	19.09	20.14	20.88	54.37	Degenerated neurons (fluoro-jade C staining)	
5xFAD + SLCP	24.03*	24.00**	7.00*	7.22*	16.50	39.37**		
% ↓ FJC + neurons by SLCP treatment	33.73	47.70	63.33	64.11	21.01	26.55		

To investigate the number of degenerating neurons in 5xFAD mice and to determine whether SLCP had any protective effects, fluoro-jade C (FJC) staining was performed on tissue from the PFC, as well as the CA1 and CA3 areas of hippocampus. An increase in percentage of degenerated neurons was observed in all these brain areas for the 5xFAD mice, in both the 6- (Fig. 2g, h) and 12-month-old (Fig. 2i, j) vehicle-treated 5xFAD mice. The SLCP treatments prevented the percentage of increased degenerated neurons in both the 6-and 12-month-old groups (Fig. 2h, j) in the PFC, in the CA1, and in the CA3 area. The degeneration was more prevalent in 12-month-old group of 5xFAD mice than for the 6-month-old groups, and CA3 area was more affected than CA1 area (Table 4).

### SLCP treatment decreased Aβ plaque load in 5xFAD mice

After 2 months of treatments, the brain sections of the 5xFAD mice were stained for Aβ plaques with curcumin, an Aβ amyloid-specific dye (Fig. 3a). The number of plaques was quantified in different brain areas in both 6- and 12-month-old 5xFAD mice receiving SLCP or vehicle. The number of Aβ plaques were significantly higher in the PFC, CA1, CA3, DG, EC, and subicular complex (morphometric data not shown) of the vehicle-treated 5xFAD mice, while treatments of SLCP prevented this increase in plaque number (Fig. 3b–d). Similarly, our Western blot data showed that Aβ levels were significantly higher (band at 60–80 kDa) in PFC and in hippocampus of both the 6- and 12-month-old and that SLCP significantly decreased these levels (Fig. 3e–g).

**Fig. 3:** SLCP inhibited Aβ plaque load and amount of Aβ in 5xFAD brain. Six- and twelve-month-old 5xFAD and age-matched control animals were treated with SLCP (100 mg/kg) or vehicle for 2 months, and their brains were perfused with 4% paraformaldehyde. Forty-micron coronal sections were made using a cryostat and were stained with for Aβ using a curcumin-based solution (1 μM, dissolved 70% methanol, 10 min) and the images were taken using a fluorescent microscope with a × 20 objective (total magnification = × 200). **a** Representative images show that curcumin binds with Aβ, similar to Aβ-specific antibody (6E10). **b** Representative images of Aβ plaques stained by curcumin in cortex, hippocampus (CA1, CA3, DG, subicular complex), and entorhinal cortex from vehicle- and SLCP-treated 5xFAD mice at both 6- and 12-months of age. **c**, **d** Morphometric analysis showed that Aβ plaques were significantly less (*p < 0.05 and **p < 0.01) in all the abovementioned areas of 5xFAD mice treated with SLCP. **e** Representative Western blot data for Aβ levels from cortical and hippocampal tissue in WT and 5xFAD mice after treatment with SLCP and probe with 6E10. **f, g** Densitometric analysis revealed that SLCP treatment significantly decreased Aβ levels in 5xFAD mice treated with SLCP in both cortical and hippocampal tissue in both 6- (**f**) and 12-month (**g**) mice. Scale bar = 100 μm and is applicable to all images. *p < 0.05, **p < 0.01 in comparison to WT + vehicle, 5xFAD + SLCP, and WT + SLCP

### SLCP treatment prevented abnormal dendritic arborization and dendritic spine morphology in the PFC, CA1, CA3, and EC of 5xFAD mice

Dendritic arborization and the number of dendritic spines are significantly affected by AD. We observed a reduction of dendritic branching, along with disorientation of apical and basal dendrites in PFC (Fig. 4a), EC (Fig. 4f), CA1 (Fig. 5a), and CA3 (Fig. 5f) pyramidal neurons in vehicle-treated 5xFAD mice in comparison to age-matched WT mice. We found that apical branches were more affected than basal branches in all these brain areas. Treatments with SLCP prevented losses in dendritic branching and sprouting.

**Fig. 4:** SLCP treatment prevented abnormal dendritic arborization and loss of dendritic spines in the PFC and entorhinal cortex of 5xFAD mice. Six- and twelve-month-old 5xFAD and age-matched control mice were treated with SLCP (100 mg/kg) or vehicle for 2 months and then their brains were extracted and stained with Golgi-Cox stain over a 2-week period. Coronal sections (120 μm) were stained with 75% ammonium solution and 1% sodium thiosulphate. Cortical pyramidal neurons (layer II-III), along with dendritic spines from apical and basal branches (primary, secondary, and tertiary) were imaged using × 40 and × 100 objectives, respectively. **a** Representative images from layer II cortical pyramidal neurons processed with Golgi-Cox stain. Note that apical and basal branches are relatively less in vehicle-treated 5xFAD mice and that SLCP treatment prevented this loss. **b, d** Representative dendritic spine images from apical and basal branches. **c, e** Morphometric data revealed that the number of dendritic spines were significantly decreased in vehicle-treated 5xFAD mice in comparison to their WT counterparts, whereas SLCP treatment mitigated these losses. **f** Representative images of layer II pyramidal neurons from entorhinal cortex. Fewer apical and basal branches were observed less in the vehicle-treated 5xFAD mice, but SLCP treatments mitigated this loss. **g, i** Representative dendritic spine images from apical and basal branches. **h, j** Dendritic spine density was significantly decreased in 5xFAD mice in comparison to WT mice, but SLCP treatment prevented much of this loss. **k** Representative images of apical and basal dendrites. **l** Representative images of primary, secondary, and tertiary dendrites from apical branch. Scale bar = 100 μm and is applicable to all images. *p < 0.05, **p < 0.01 in comparison to WT + vehicle, 5xFAD + SLCP, and WT + SLCP

**Fig. 5:** SLCP treatment partially preserved dendritic arborization and dendritic spine number in hippocampus of 5xFAD mice. After 2 months of treatment with SLCP (100 mg/kg), the brains of the 6- and 12-month-old 5xFAD and age-matched control mice were processed using Golgi-Cox stain for 2 weeks. Coronal sections (120 μm) were stained with 75% ammonium solution and 1% sodium thiosulphate. CA1 and CA3 neurons and dendritic spines from apical and basal branches (primary, secondary, and tertiary) were imaged using 40x and  100x objectives, respectively (Olympus). **a, f** Representative images of CA1 and CA3 pyramidal neurons showed a decreased number of apical and basal branches in vehicle-treated 5xFAD mice in comparison to WT and SLCP-treated mice. **b, d** Representative dendritic spine images from apical and basal branches. **c, e** Morphometric data revealed that the number of dendritic spines in CA1 neurons were significantly decreased in vehicle-treated 5xFAD mice in comparison to WT and SLCP-treated mice. **g, i** Representative dendritic spine images from CA3 apical and basal branches, respectively. **h, j** Morphometric analyses showed that the number of dendritic spines were significantly decreased in vehicle-treated 5xFAD mice in comparison to their WT counterparts, and to SLCP-treated 5xFAD mice. Scale bar = 100 μm and is applicable to all images. *p < 0.05, **p < 0.01 in comparison to WT + vehicle, 5xFAD + SLCP, and WT + SLCP

#### Dendritic spine number in PFC

The number of dendritic spines was significantly less in PFC neurons in the vehicle-treated 5xFAD mice in comparison to WT mice, in both primary and secondary apical branches (Fig. 4b, c). Similarly, percentage of dendritic spines in primary and secondary basal dendrites of vehicle-treated 5xFAD mice were also significantly decreased in comparison to age-matched WT mice (Fig. 4d, e). In contrast, SLCP treatments in both 6- and 12-month-old 5xFAD mice significantly preserved the dendritic spine density in both apical and basal dendritic branches (Fig. 4b–e) (Table 5). In addition, 12-month-old 5xFAD mice had fewer dendritic spines number in comparison to 6-month-old vehicle-treated 5xFAD mice. Similar trends were observed in percentage changes of dendritic spine number in the case of tertiary apical and basal branches (data not shown).

**Table 5:** Percentage reduction of dendritic spine density in PFC, CA1, CA3, and EC areas in vehicle-treated 5xFAD and 5xFAD treated with SLCP in comparison to age-matched WT mice. *6-m* 6-month-old, *12-m* 12-month-old. *p < 0.05 and **p < 0.01 when compared with vehicle-treated 5xFAD mice

Areas	Groups	Apical branch				Basal branch			
		Primary branch		Secondary branch		Primary branch		Secondary branch	
		6-m	12-m	6-m	12-m	6-m	12-m	6-m	12-m
PFC	5xFAD + vehicle	47.70	66.45	50.83	61.93	42.34	61.48	62.13	56.87
	5xFAD + SLCP	21.66**	30.32**	16.71**	31.55**	27.35**	27.48**	30.06	17.09**
CA1	5xFAD + vehicle	41.88	48.71	45.13	58.58	24.64	47.00	30.86	61.96
	5xFAD + SLCP	29.22	20.62**	8.91**	33.18**	8.09**	31.50*	12.67*	29.67**
CA3	5xFAD + vehicle	57.03	67.52	53.49	71.12	30.86	72.84	31.32	60.60
	5xFAD + SLCP	33.76**	43.92**	38.10*	39.42**	9.25	24.85**	14.37	20.12**
EC	5xFAD + vehicle	45.67	48.50	43.72	49.18	37.87	45.12	35.99	62.46
	5xFAD + SLCP	28.86**	37.78	21.24*	35.20*	20.49*	1.65**	16.21*	31.80**

#### Dendritic spine number in entorhinal cortex

The number of dendritic spines in EC, another vulnerable area affected by AD, was reduced in 5xFAD mice in comparison to WT mice, whereas SLCP treatments partially preserved their normal levels (Fig. 4f, j). In contrast, differences in dendritic spine number in primary basal branch in 6-month-old 5xFAD mice compared to WT were minimal, whereas in the case of 12-month-old group of mice, the percentage of dendritic spine losses were decreased in comparison to WT mice (Table 5). Similarly, percentage changes of dendritic spine number in tertiary apical and basal branches were like those observed in the primary and secondary branches (data not shown). Percentage loss of dendritic spine was larger for in 12-month-old 5xFAD mice in comparison to 6-month-old groups (Table 5).

#### Dendritic spine number in CA1 area

A significant decrease in spine number in CA1 area in the hippocampus was observed in the vehicle-treated 5xFAD mice, with SLCP treatments significantly preserving the number of dendritic spines in both apical and basal branches (Fig. 5b–e). Percentage reduction of dendritic spine number was significantly higher in 12-month-old vehicle-treated 5xFAD mice in comparison to 6-month-old mice (Table 5). The percentage loss of dendritic spines in the tertiary apical and basal branches has shown a similar pattern (data not shown). A significant number of varicosities were observed in 5xFAD mice, which was reduced by SLCP treatment (data not shown).

#### Dendritic spine number in CA3 area

A significant reduction of dendritic spines in the CA3 area of hippocampus was observed in both 6- and 12-month-old vehicle-treated 5xFAD mice in comparison to age-matched WT mice (Fig. 5f–j). Twelve-month-old 5xFAD mice showed significantly more loss of dendritic spine in comparison to 6-month-old mice. However, no significant differences in dendritic spine number were observed between primary and secondary branches of both apical and basal branches (Table 5). In contrast, SLCP treatments significantly prevented these losses in both the apical and basal branches in 12-month-old groups of mice (Fig. 5h, j) (Table 5). Although the dendritic spine number was preserved in the CA3 apical branch of 6-month-old mice, no significant differences between vehicle-treated 5xFAD and 5xFAD + SLCP groups were observed in this structure (Fig. 5i, j). Overall, dendritic spine number was more affected in CA3 area in comparison to CA1 area in both 6- and 12-month 5xFAD mice (Figs. 4 and 5).

### SLCP preserved synaptophysin and PSD95 levels in cortex and hippocampal subfields in 5xFAD mice

After 2 months of SLCP treatment, brain sections were immunolabeled with synaptophysin and PSD95 antibodies. We observed that the immunofluorescent signal for synaptophysin was comparatively less in vehicle-treated 5xFAD mice in all the brain areas (PFC, and the CA1 and CA3 subfields of hippocampus) in both 6- and 12-month-old mice, while SLCP treatment showed partial preservation of these signals (Fig. 6a, b). Our Western blot data analysis revealed that relative to WT mice, synaptophysin levels were significantly decreased in vehicle-treated 5xFAD mice by 35.03% and 19.91% in the cortex in the vehicle-treated 6- and 12-month-old groups, respectively and 32.86% and 35.79% in the hippocampus of 6- and 12-month-old vehicle-treated 5xFAD mice, respectively (Fig. 6e–h). In contrast, SLCP-treated 5xFAD mice had significantly lower decrease in these levels, with only 25.01% and 45.01% in the cortex of 6- and 12-month-old mice, respectively, and 9.16% and 17.34% in the hippocampus of 6- and 12-month mice (Fig. 6e-f, i, j), respectively.

**Fig. 6:** SLCP treatment partially preserved synaptophysin and PSD95 levels in the PFC and hippocampus of 5xFAD mice. Six- and 12-month-old 5xFAD and age-matched controls were treated with SLCP (100 mg/kg) for 2 months and then their brains were extracted, sectioned coronally at 40 μm, and stained with anti-synaptophysin and PSD95 antibodies. Images were taken using a fluorescent microscope at  4x0 (total magnification =  400x). **a, b** The vehicle-treated 5xFAD mice showed a decrease in synaptophysin fluorescent signals in the cortex, as well as the CA1, and CA3 areas of the hippocampus when compared to WT and SLCP-treated mice. **e–h** Western blot data from cortical and hippocampal tissue showed that synaptophysin was significantly reduced in vehicle-treated 5xFAD mice and that SLCP treatment prevented much of these losses. Scale bar= 100 μm and applicable to all other images. **c, d** Immunofluorescent intensity was decreased in vehicle-treated 5xFAD mice in comparison to WT mice, but SLCP treatments moderately preserved these levels in all three of the brain regions sampled. **e, f** and **i, j** Western blot data from cortical and hippocampal tissue showed that PSD95 levels were significantly reduced in vehicle-treated 5xFAD mice and that SLCP treatment partially preserved these levels. Scale bar indicates 100 μm and applicable to all images. *p < 0.05, **p < 0.01 in comparison to WT + vehicle, 5xFAD + SLCP, and WT + SLCP. Scale bar = 100 μm for all images.

Similarly, we also observed apparent decreased fluorescent signals for PSD95 in vehicle-treated 5xFAD mice, with SLCP treatments moderately preserving this signal (Fig. 6c, d). Our Western blot data also indicated that the levels of PSD95 were significantly lower in cortex by 64.17% and 49.61% in the 6- and 12-month-old 5xFAD mice, respectively and 40.41% and 37.83% in hippocampus of the 6- and 12-month-old vehicle-treated 5xFAD mice, respectively, when compared to WT mice. Importantly, SLCP treatment significantly reduced these losses with 49.61% and 4.32% in cortex of the 6- and 12-month-old 5xFAD mice, respectively, and by 14.84% and 13.65% in the hippocampus of the 6-and 12-month-old 5xFAD mice, respectively, when compared to 5xFAD mice treated with vehicle (Fig. 6e–f, i, j). Although we did not find any region-specific differences in the levels of synaptophysin and PSD95 after SLCP treatment, we did observe a greater preservation of these two-protein markers in 6-month-old groups in comparison to 12-month-old groups of mice.

### SLCP treatment preserved dendritic spine signaling markers in cortex and hippocampus of 5xFAD mice

Western blots were performed on cortical and hippocampal tissue from the 6- and 12-month-old mice using different postsynaptic signaling antibody markers (Fig. 7a–g). Shank (Fig. 7b), Homer (Fig. 7c), and Drebrin (Fig. 7d) levels were significantly reduced in vehicle-treated 5xFAD mice, in comparison to WT mice, whereas SLCP-treated 5xFAD mice had partially preserved levels. Similarly, we found a significant reduction in total CREB and pCREB levels in 5xFAD mice and SLCP treatment significantly preserved those levels (Fig. 7f–g). In contrast, we did not find any significant changes of Kalirin-7 levels among all these groups (Fig. 7a, e).

**Fig. 7:** SLCP treatment preserved dendritic spine-signaling markers in PFC and hippocampus of 5xFAD mice. Six- and 12-month-old 5xFAD and age-matched control mice were treated with SLCP (100 mg/kg) for 2 months and then their brains were extracted, and cortical and hippocampal tissue homogenates were processed for Western blot analyses using antibody probes for selected proteins. **a** Representative Western blots from cortical and hippocampal tissue in 5xFAD mice, with or without treatment with SLCP. **b–g** Optical densitometric measures from 3 to 4 blots from each protein sample were made. Note that Shank, Homer, Drebrin, pCREB, and total CREB were significantly reduced in vehicle-treated 5xFAD mice and that SLCP treatments partially preserved these levels. *p < 0.05 in comparison to WT + vehicle, 5xFAD + SLCP, and WT + SLCP

## Discussion

Metabolic dysfunction, increase neuroinflammation, and disturbances of protein homeostasis are associated with increased neurodegeneration, synaptic loss, and memory impairment in AD [51]. Therefore, decreasing misfolded protein loads and preventing synaptic loss are viable options for preserving cognitive function in AD [52]. In the present study, we have investigated the effects of chronic administration of SLCP in 5xFAD mice in different brain areas on (i) neuronal morphology, (ii) neurodegeneration, (iii) amyloid plaque burden; (iv) dendritic spine morphology; (v) the pre-and postsynaptic signaling markers; and (vi) on neurobehavioral outcomes. We observed a significant preservation of dendritic spine morphology and pre- and post-synaptic protein markers in different brain areas, along with partial protection against cognitive dysfunction in 5xFAD mice after treatment with SLCP.

Several anti-amyloid, anti-inflammatory drugs, and small molecules have been tested as potential treatments for AD. However, none of these have translated into successful treatments in clinical AD trials [53]. Curcumin, a potent anti-amyloid, anti-inflammatory, anti-oxidant natural polyphenol, has shown promising effects as an AD therapy [20, 21, 23–26, 29, 30]. Because of its unique physicochemical, anti-amyloid, anti-inflammatory, and anti-oxidant properties, Cur is considered a relatively safe treatment for AD [54–57]. Unfortunately, the lipophilic and hydrophobic nature of this natural polyphenol reduces its solubility and bioavailability, which limits its clinical utility [56, 58]. However, the use of Cur-coated solid lipid particles (SLCP) shows significant promise in providing greater neuroprotection in animal models [18, 29] and clinical trials of AD [33]. Our previous studies suggest that SLCP is a more effective anti-amyloid, anti-inflammatory, and neuroprotective agent than natural curcumin [29]. Although the specific procedures for making the SLCP used are proprietary to Verdure Sciences and we did not compare the activities and bioavailability of SLCP with other Cur formulations such as Theracurmin or curcugreen, the available information suggests that there are several advantages to use SLCP (LongVida) over other Cur formulations, including Theracurmin or curcugreen. The SLCP we used can tolerate harsh digestive pH condition and is not being destroyed by the acidic environment of stomach. In addition, the small particle size of the LongVida Cur can easily passage across the membrane of the intestine. It provides a unique coating of highly purified fatty acids and phospholipids that surrounds the Cur molecules and enables it to be transported into the lymphatic system rather than the circulatory system. Because it bypasses the liver, SLCP has reduced exposure to metabolic enzymes and remains in a free form. Although the "theracurmin", a water-dispersible formulation and the "curcugreen" which contains 86% curcuminoids and 7-9% ar-tumarone, an essential oil of turmeric extract are highly bioavailable, the bioavailability of SLCP (LongVida) is 285 times greater, has 65 times the peak plasma levels, and lasts seven times longer than standard Cur [24], suggesting that its properties compared favorably with other curcumin derivatives, including Theracurmin [59] or curcugreen. In the present study, we have investigated whether SLCP can protect against synaptic loss, especially on dendritic arborization, postsynaptic signaling proteins, and neurobehavioral impairments in the 5xFAD mouse model of AD.

Initially, we compared the anti-amyloid capability of natural Cur and SLCP formulation using dot blot assay (S2). We used synthesized Aβ42 peptide (10 μM) and allowed it to aggregate with or without Cur or SLCP. We clearly observed more inhibition of aggregation in Aβ42 oligomers and fibrils treated with SLCP than with Cur (S2). This might be due to greater affinity and interactions of SLCP (because of lipid content) with C-terminal hydrophobic fragment of Aβ, as observed previously [60, 61]. Interestingly, we found that low (1 nM) concentrations of Cur were able to inhibit Aβ42 oligomers and fibrils in vitro, suggesting that very negligible amounts of Cur are required for halting Aβ assembly [21]. Based on these findings and our previous observations [21, 29], we decided to use SLCP as a potential therapy in 5xFAD mice. After 2 months of oral gavage, we found a significant decrease in Aβ plaque burden in several brain areas, such as PFC, EC, CA1, CA3, DG, and subicular complex (Fig. 3a-d). In addition, our Western blot data provided further evidence that SLCP can reduce Aβ plaque load (Fig. 3e–g), suggesting that the lipid-coated SLCP facilitates its permeability into the brain tissue and inhibits amyloidogenic pathways, either by reducing Aβ production or preventing its aggregation [60]. However, we did not measure the level of free Cur in the SLCP-treated mice brain tissue, when we injected SLCP (100 mg/kg) for 5 consecutive days, intraperitoneally, and observed curcumin labeled Aβ plaques in cortical and hippocampal tissue (S5), which confirmed that SLCP penetrated brain tissue [21, 29]. In addition, we previously found that 300–400 nM of free Cur accumulates in the brain tissue and 2–3-fold more is found in the plasma, when mice were given a dose of ~ 1.25 mg/day or 83 mg/kg [23, 24]. In addition, these findings were also supported by a clinical trial in AD patients [33] with the same formulation, suggesting that SLCP is highly permeable to brain tissue and capable of reducing AD pathologies.

We also investigated whether SLCP treatments decreased Aβ load and preserved neuronal morphology in affected areas of the 5xFAD brain. We used cresyl violet (CV) and fluoro-jade C (FJC) stains in both paraffin-embedded and cryostat-sectioned tissue to investigate overall neuronal morphology and degenerated cells, respectively. Our morphometric data revealed that SLCP treatment significantly reduced the number of pyknotic cells (Fig. 2a–e) and reduced the number of degenerated cells (Fig. 2g–j) in all the sampled brain areas of the 5xFAD mouse brain. These findings paralleled findings of decreased Aβ plaque burden in SLCP-treated 5xFAD mice, suggesting SLCP may have an inhibitory role on Aβ production, as reported by many other investigators [60–62]. We observed a greater degenerative change in the CA3 region of the hippocampus in comparison to CA1 neurons, a finding which differs from that of Padurariu and colleagues [63]. This discrepancy may be because Padurariu and colleagues used human AD patients and we used 5xFAD mice which may have differential mechanisms involving region-specific neuronal death, a possibility which needs further investigation. In addition, we also found that EC neurons (layer II) were more affected than those in the PFC area (layer II-III). These findings also correspond with our CV (Fig. 2a–d) and FJC (Fig. 2g–j) morphometric data, suggesting greater vulnerability of EC and over PFC neurons in 5xFAD mice. Recently, Yang and colleagues [64] reported that the entorhinal cortex (EC) is one of the most vulnerable brain regions in the early stages of AD. Because the EC innervates the CA1, its early damage during the progression of AD likely leads to a selective degeneration of more CA1 neurons and CA3 in AD mice [65], which supports our current findings.

Synaptic failure, especially the loss or degeneration of dendritic spines (DS), is closely associated with synaptic dysfunction, cognitive decline, and memory loss in AD [54]. Accumulation of misfolded Aβ species, especially diffusible oligomers, is closely linked with dendritic spine dysfunction in AD [55, 56]. Therefore, prevention of dendritic spine loss and restoration of synaptic signaling proteins could be a viable approach to preserve cognitive function in AD. As a semi-autonomous compartment of excitatory neurons, dendritic spines regulate Ca^++^ levels and are involved in synaptic signaling, as well as in development of long-term potentiation (LTP), which is a putative molecular basics for learning and memory [64, 66]. Several investigators reported numerous alterations have been observed in early stages of the AD brain, including dendritic arborization, and loss of dendritic spines, which correlate with cognitive dysfunction [8, 67, 68]. Interestingly, the loss of dendritic spines was more profoundly observed around the Aβ plaques at 12 months of age (Table 5) in the 5xFAD mouse brain [69].

Collectively, these observations prompted us to investigate whether SLCP has any role for preserving dendritic arborization and dendritic spine density in 5xFAD mice, especially in the most affected brain areas of this AD mouse model. We studied dendritic arborization and spine density from primary, secondary, and tertiary branches of both apical and basal dendrites in PFC (layer II), CA1, CA3, and EC (layer II) neurons from 6- and 12-month-old 5xFAD mice by Golgi-Cox stain after treatment with SLCP or vehicle. We observed a marked decrease in the number of dendritic branches from the pyramidal neurons of PFC and EC (Fig. 4), CA1 and CA3 areas of hippocampus (Fig. 5). We quantified the number of dendritic branches and found that they were significantly lower in 5xFAD mice, but that SLCP treatment mitigated this loss (data not shown). Although we did not quantify the length of different dendritic branches using Sholl analysis, the dendritic length appeared to be smaller in the vehicle-treated 5xFAD-vehicle-treated mice when compared with age-matched WT controls and to SLCP-treated 5xFAD mice. When we analyzed the spine density from different brain areas, we found a significant reduction of both apical and basal dendritic spines in in PFC, CA1, CA3, and EC areas in both 6- and 12-month-old 5xFAD mice (Figs. 4 and 5). Interestingly, we found a large reduction in the case of 12- versus 6-month-old 5xFAD mice. Furthermore, vehicle-treated 5xFAD mice of both 6- and 12-month-old showed lots of varicosities and ectopic spines, especially in primary and secondary apical dendritic branches, which was relatively less observed in SLCP-treated 5xFAD mice. In addition, we also observed less cup- or mushroom-shaped dendritic spines in 5xFAD mice compared to SLCP-treated groups, indicating overall preservation of mature spines by SLCP. However, we did not find region-specific differences in loss of spine density among any of the groups. One reason for this might be that we did not count dendritic spine number using unbiased stereology, which may have provided a more accurate means of comparisons. However, we took proper precautions to avoid biases in our counting by selecting dendrites that were only 2–3 μm for primary, 1–2 μm for secondary, and ≤ 1 μm for tertiary branches, to avoid counting of hidden spines beneath the dendritic shaft. In addition, we did not categorize different types of dendritic spines in this study. For example, thin spines have the highest incidence of remodeling, whereas mushroom spines have the lowest capability for remodeling and are more affected in 5xFAD mice. Therefore, further investigations are needed to confirm and extend these findings, especially in the context of the dose and duration of curcumin treatments.

Synaptic loss is one of the primary causes for Aβ accumulation and cognitive dysfunction in AD [70]. Loss of synaptophysin [71] and PSD95 are associated with degeneration of dendritic spines and have been shown to be directly correlated with impaired recognition memory and spatial memory [72]. Therefore, we have studied pre- and post-synaptic protein markers (Figs. 6 and 7) in this study. Our Western blot data suggest that SLCP preserved levels of synaptophysin, PSD95, and other dendritic spine-signaling proteins, such as Shank, Homer, and Drebrin levels (Fig. 7). Recently, natural curcumin has been shown to increase synaptophysin levels in brains of 5xFAD mice [59, 61, 73], and these observations support our findings. Similarly, PSD95 levels were preserved by SLCP treatment in 5xFAD mice (Fig. 6c, d, e, f, i, j), which, again, supports our findings [59, 74]. Furthermore, cyclic adenosine monophosphate (cAMP) response element-binding protein (CREB) signaling pathway is very important in learning and memory and is significantly impaired in 5xFAD mice, as well as in Aβ-infused models, of AD. We found moderately improved levels of pCREB and total CREB after treatment with SLCP (Fig. 7a, f, g), which was also observed by Zhang and colleagues in an animal model of AD after Cur treatment [73]. Furthermore, Shank, Homer, Drebrin, and Kalirin-7 are also linked with PSD95, and loss of these proteins causes impairment of postsynaptic signaling, as observed in different neurological diseases, including AD [75]. We found that SLCP treatment improved their levels (except for Kalirin-7) in 5xFAD mice, suggesting SLCP has an ameliorating role in the dendritic spine-signaling pathway, as reported by many other researchers using curcumin treatment. Overall, partial restoration of these marker proteins by SLCP treatment in 5xFAD mice may be due to restoration of spine density, which may in turn be due to decreased Aβ load (Fig. 7) and decreased neuroinflammation, as we observed in our previous studies [29] (Fig. 8).

**Fig. 8:** Schematic diagram showing possible mechanism of synaptic preservation and improvement of cognitive function in 5xFAD after SLCP treatment

Several studies suggest that daily intake of curcumin may have ameliorative behavioral effects, especially for improving learning, memory, and attention in normal individuals [76]. Therefore, we attempted to investigate the effects of SLCP on behavioral measures, including AD-associated cognitive impairment. We used an open-field test and counted number of fecal boli as a measure of anxiety levels, following treatment, and found that the 5xFAD mice produced more boli during pre-treatment trial, but no between-group differences were observed during post-treatment trials. However, we did observe a persistent hyperactivity in both 6- and 12-month-old 5xFAD mice (S3C and D), which was ameliorated by SLCP treatment. Results from our NOR task, which measures recognition memory, commonly impaired in AD patients [77], indicated a significant decrease in both the discrimination index (S4C) and the exploration index (S3B). We observed that 5xFAD mice treated with SLCP explored the novel object more than did vehicle-treated 5xFAD mice at 12 months of age, suggesting that SLCP treatment spared recognition memory in aged 5xFAD mice. Because spatial memory is significantly impaired in AD patients, we performed Morris water maze (MWM) task and found a significant increase in escape latency and path length to find the hidden platform in the 12-month-old vehicle-treated 5xFAD mice, relative to SLCP-treated mice which found the hidden platform faster during the last 2 days of training session (Fig. 1). In addition, during the probe trial, SLCP-treated 5xFAD mice spent less time to enter to the target quadrant and kept their mean distance closer to the target (previous position of the platform)  compared to the vehicle-treated 5xFAD mice, suggesting SLCP protects against spatial memory deficits in 5x FAD mice. Recently, Kim and colleagues also found that a modified formulation of Cur ameliorated cognitive dysfunction in 5xFAD mice by improving synaptic function [59]. Smilarly, we and other also reported that SLCP have beneficial effects in mouse model of Huntington's disease [78, 79]  Thus, our findings confirm earlier findings and extend previous research showing the ameliorating effects of SLCP in counteracting both impaired recognition memory and spatial memory dysfunction in an AD mouse model by normalizing synaptic function.

## Conclusions

Taken together, our findings suggest that SLCP offers neuroprotective effects by decreasing amyloid plaque load, preserving dendritic spine arborization, and protecting synaptic signaling proteins, mitigating the cognitive and behavioral deficits in 5xFAD mice. Further extension of these results has important clinical implications, especially those where anomalies in dendritic spines are observed, such as in many neurodegenerative diseases, including AD.

### Limitations

(i) We did not measure the amount of free Cur in the SLCP-treated mice brain tissue after 2 months of treatment in the present study. However, in our previous study, we measured curcumin levels by HPLC/mass spectroscopy with same formulation with same dose and duration and we found ~ 300–400 nM of free curcumin accumulates in the brain tissue and 2–3-fold more is found in the plasma, when mice were given a dose of ~ 1.25 mg/day or 83 mg/kg [24]. (ii) For histology, immunohistochemistry, and Western blot analyses, we have used 3 mice per group for each study. (iii) We did not quantify the length of different dendritic branches using Sholl analysis. Also, due to unavailability of stereology software, we did not count the dendritic spine number using unbiased stereology, which may have provided a more accurate means of comparisons.

## Supplementary Information

**Additional file 1: S1.** Schematic diagram showing experimental design, treatment paradigm.

**Additional file 2: S2.** SLCP inhibited Aβ-aggregation more efficiently than natural curcumin. Synthesized Aβ42 (10 μM) was disaggregated with hexafluorisopropanol and dissolved in phosphate buffer saline (PBS, 0.1 M, pH 7.4) and allowed to aggregate in presence or absence of different concentrations of natural curcumin and SLCP, after which a dot-blot analysis was performed. About 10 μl of peptide solution was spotted on PVDF membrane and probed with Aβ fibril (6E10, OC) and oligomer specific (A11) antibodies. A-F: SLCP showed greater inhibition of Aβ42 aggregation after 24 h (A and B), 48 h (C and D), and 72 h (E and F) of incubation in comparison to natural curcumin (Cur). G-H: Aβ42 oligomers formation was also inhibited more efficiently by SLCP than Cur after 8 h of incubation. I-L: Similarly, SLCP inhibited Aβ42 fibril formation more efficiently than Cur after 24- (I-J) and 48 h (K-L) of incubation. In addition, lower concentrations (1–100 nM) of both SLCP and Cur inhibited Aβ42 aggregation more efficiently than higher concentrations did. Results represented as mean ± SEM from three independent experiments. *p < 0.05, **p < 0.01 in comparison to Aβ42 treated with vehicle.

**Additional file 3: S3.** Effects of SLCP on spontaneous motor activity and fecal boli count in the open-field task. The open-field test was used to access overall activity of the mice, both pre-and post-treatment. A and B: No significant between-group differences were observed in speed (cm/sec) during movements for both pre- and post-treated mice in either age group. C and D: Prior-to treatment, the 5xFAD mice traveled significantly more distance than WT + Vehicle, but SLCP treatment prevented this hyperactivity in both age groups. E-F: Total number of fecal boli count in both the 6-month-old (E) and 12-month-old (F) group of animals indicated significant increases in 5xFAD mice prior to treatment, but no between-group differences were observed during post-treatment testing. *p < 0.05 in comparison to WT + Vehicle. # p < 0.05, changes with all post-treatment, except 5xFAD + SLCP mice, † p < 0.05, compared with all post-treated groups.

**Additional file 4: S4.** Effects of SLCP on recognition memory in the novel-object-recognition task. A-C: Six- and twelve-month-old 5xFAD and age-matched control mice were tested on the novel object recognition (NOR) task after treatment with SLCP (100 mg/kg) for 2 months. A: The 12-month-old 5xFAD mice spent less time exploring the novel object than WT mice, but this recognition deficit was not observed in 5xFAD mice treated with SLCP. The exploration index (B) was also significantly reduced in the 12-month-old 5xFAD, the discrimination index (C) was decreased in both 6- and 12-month-old 5xFAD mice, but not in 5xFAD mice treated with SLCP. *p < 0.05 in comparison to WT + Vehicle, 5xFAD + SLCP and WT + SLCP-treated mice.

**Additional file 5: S5.** Curcumin cross blood brain barrier and reach to brain tissue. Twelve-month-old 5xFAD mice was injected with SLCP (100 mg/kg) for 5 days intraperitoneally. Brain was perfused with PBS and 4% paraformaldehyde and coronal section was made by cryostat and probe by 6E10 and appropriate secondary antibody conjugated with Texas-red. Images were taken in fluorescence microscope using a 40x objective. Curcumin premetallized to brain tissue, labeled with amyloid plaques. Arrow indicates amyloid plaque. A: cortical area; B: dentate gyrus of hippocampus. C: Colocalization of curcumin with 6E10 in intracellular Aβ in 12-month-old 5xFAD mouse cortical neurons. Red: 6E10; green: curcumin, blue: DAPI. Scale bar = 250 μm (upper) and 50 μm (lower).

## Data Availability

The data generated and/or analyzed in this are included in the article and the data and materials are available from the corresponding authors on reasonable request.

## Abbreviations

AD: Alzheimer’s disease
Cur: Curcumin
SLCP: Solid lipid curcumin particles
FAD: Familial Alzheimer’s disease
PFC: Prefrontal cortex
EC: Entorhinal cortex
SC: Subicular complex
FJC: Fluoro-jade C
GC: Golgi-Cox
PSD95: Postsynaptic density protein 95
CREB: Cyclic adenosine monophosphate element-binding protein
NOR: Novel object recognition
MWM: Morris water maze
OF: Open-field
Aβ: Amyloid beta protein
FDA: Food and drug administration
PVDF: Polyvinylidene difluoride
DAPI: 4′,6-Diamidino-2-phenylindole
BCA: Bicinchoninic acid
TBS-T: Tris-buffered saline with Tween 20
HRP: Horseradish-peroxidase
APP: Amyloid precursor protein
IACUC: Institutional Animal Care and Use Committee
BW: Body weight
IF: Immunofluorescent
WB: Western blot
FO: Familiar object
TN: Time in contact withnovel object
TF: Time in contact with familiar object
DI: Discrimination index
PBS: Phosphate-buffered saline
CV: Cresyl violet
NGS: Normal goat serum
RIPA: Radioimmunoprecipitation assay
SDS-PAGE: Sodium dodecyl sulfate polyacrylamide gel electrophoresis
ANOVA: Analysis of variance
HSD: Honestly significant difference
LTP: Long-term potentiation
cAMP: Cyclic adenosine monophosphate
